# Estimation of Breathing Rate with Confidence Interval Using Single-Channel CW Radar

**DOI:** 10.1155/2019/2658675

**Published:** 2019-03-28

**Authors:** I. Nejadgholi, H. Sadreazami, Z. Baird, S. Rajan, M. Bolic

**Affiliations:** ^1^School of Electrical Engineering and Computer Science, University of Ottawa, Ottawa, ON, Canada; ^2^Department of Systems and Computer Engineering, Carleton University, Ottawa, ON, Canada

## Abstract

Breathing rate monitoring using continuous wave (CW) radar has gained much attention due to its contact-less nature and privacy-friendly characteristic. In this work, using a single-channel CW radar, a breathing rate estimation method is proposed that deals with system nonlinearity of a single-channel CW radar and realizes a reliable breathing rate estimate by including confidence intervals. To this end, time-varying dominant Doppler frequency of radar signal, in the range of breathing rate, is extracted in time-frequency domain. It is shown through simulation and mathematical modeling that the average of the dominant Doppler frequencies over time provides an estimation of breathing rate. However, this frequency is affected by noise components and random body movements over time. To address this issue, the sum of these unwanted components is extracted in time-frequency domain, and from their surrogate versions, bootstrap resamples of the measured signal are obtained. Accordingly, a 95% confidence interval is calculated for breathing rate estimation using the bootstrap approach. The proposed method is validated in three different postures including lying down, sitting, and standing, with or without random body movements. The results show that using the proposed algorithm, estimation of breathing rate is feasible using single-channel CW radar. It is also shown that even in presence of random body movements, average of absolute error of estimation for all three postures is 1.88 breath per minute, which represents 66% improvement as compared to the Fourier transform-based approach.

## 1. Introduction

Breathing rate is one of the four vital signs. Breathing rates may increase with fever, stress, or some medical conditions. Prolonged increased breathing rate is a cause of concern; hence, it is important to measure breathing rate. Normal breathing rates for an adult person at rest ranges from 12 to 16 breaths per minute.

In order to measure breathing rate, one may use contact-based method such as respiratory inductive plethysmography (RIP) bands. Such bands are used for sleep tests despite the discomfort to the subjects. There are several instances where such a band cannot be used. For instance, in the case of burn victims, it is not possible to use a band. In emergency departments, when patients arrive, it may not be possible to use a band to estimate breathing rate. Remote measurements are preferred in such cases. In senior's home, it is preferable to monitor breathing without the need to wear devices. In addition, correctional institutions are looking to adopt a nonobtrusive method for monitoring the vital signs of inmates, especially because it is a privacy-friendly technology compared to cameras. In addition, depending on the frequencies used for radars, it is possible to obtain both heart rate and breathing rate using a single sensor which may not be possible with RIP.

Radar has recently attracted much attention as a promising device for breathing rate monitoring, mainly because of its contact-less, privacy-friendly, and relatively safe properties [1–3]. Video cameras, as an alternative choice, have been used for contact-less monitoring of vital signs. However, cameras invade privacy and their performance is highly affected by the amount of light in the monitored space [4, 5] and pose of the subjects.

Continuous wave (CW) radar systems have widely been used for vital sign monitoring due to their low power consumption and simple radio architecture [6, 7]. This radar has also been used to see through-wall a human skeletal figure [8] and localize a small number of colocated people [9]. In such radar systems, a single-frequency signal is transmitted and signals reflected off the subjects are received. The received signal is modulated by the movements of the chest based on the Doppler principle. Most of these works have focused on the two-channel CW radar for vital sign monitoring with less attention to the effect of random body movements. In the proposed method, we employ a single-channel CW radar to estimate the vital signs, where the subjects are moving their body parts randomly.

When CW radar is used, the information of micromovements of chest and abdomen are concealed in the phase of the received signal. For small movements, i.e., the amplitude of displacement is much smaller than the wavelength of transmitted signal, the signal can be approximated by its phase, referred to as linear approximation [10]. On the other hand, in the case of larger displacements of chest and abdomen which depend on the anatomy of the subject and the type of breathing and posture, the linear approximation does not hold anymore especially when the wavelength of radar is small (<2 cm). In this case, multiple harmonics of breathing as well as intermodulations between heart rate and breathing rate are produced [11], which affect the accuracy of breathing rate estimation obtained through Fourier analysis. One possible solution to address the nonlinearity of a single-channel Doppler radar is by using a quadrature radar architecture. Since the vital sign signal is a low-frequency signal, the two output channels of the quadrature radar can be used for either complex signal demodulation [12] or arctangent demodulation [13] to calculate the total Doppler phase shift. It is known that the Doppler phase shift is directly proportional to the displacements of chest. Besides dealing with nonlinearity of the signal, integration of two channels in the architecture of CW radar can offer solutions to several challenges of vital sign monitoring such as null point effect and effect of random body movements [14–17].

In this work, breathing rate is estimated by using a single-channel CW radar and applying time-frequency analysis instead of Fourier transform. The proposed method is evaluated in a real situation, where nonlinearity, null point effect, and random body movements are considered. Multiple subjects are monitored in different postures, namely, lying, sitting, and standing, at different distances from the radar with or without random movements of body. There have been few works on cancellation of random movements of body. In [18], an antiphase signal generator was used to reduce the effect of random body movements. In [13], a phase-diversity Doppler radar was introduced that utilized three antennas, one for transmitting and the other two for receiving. The receiving antennas were isolated by half of a wavelength. In [19], the center estimation algorithm was proposed to resolve the issue of random body movements. Self-injection-locked radar was proposed in [20] to cancel body movements. In [21], empirical mode decomposition was applied to cancel only the sensor movement and not the random body movements. However, all these works used both in-phase and quadrature channels and their solutions generally resulted in an increase in system complexity, cost, and power consumption. It should be noted that so far, the estimation of vital signs, where the subject is moving their body parts randomly, has not been considered with simple-structured single-channel CW radar.

Velocity of movements of chest and abdomen changes periodically over time due to breathing. This time-varying velocity translates into time-varying Doppler frequency of reflections received by the single-channel CW radar. However, other movements of the subject can contribute to frequency modulations around the main Doppler shift that are commonly referred as micro-Doppler modulations [22]. These micro-Doppler signatures in time-frequency domain have already been used to perform classification [23, 24]. This idea has also been used to estimate vital signs during walking [25].

To estimate the breathing rate, in this work, a sequence of dominant frequencies of the signal over time in the range of breathing is extracted and used to estimate the breathing rate. The bootstrap resampling method is used to support the estimation with a confidence interval, since we are dealing with a single-channel CW radar signal in which extracted micro-Doppler shifts may be affected by movements of body and null point effect.

The paper is organized as follows.  Section 2 presents the model of reflected radar signal from a human subject using a single-channel CW radar and presents the challenges of estimating breathing rate using Fourier transform.  Section 3 presents the proposed estimation method and also discusses the bootstrap resampling method used to estimate confidence interval of breathing rate.  Section 4 presents the experimental setup and the data collection procedure.  Section 5 presents a discussion of the results. Finally, Section 6 concludes the paper.

## 2. Modeling and Simulation of Single-Channel Radar Signal

During our experiment, in order to have the entire room covered, the radar is mounted on the wall.  Figure 1 shows a scenario in which a stationary person is in front of the radar. The transmitting and receiving antennas are colocated. The transmitter transmits a radar signal that is a continuous wave which is intercepted by the subject. Movements of chest, abdomen, and heart cause Doppler shift in the frequency of the returned radar signal. At the receiver, the transmitted signal is delayed and correlated with the received signal. A low-pass filter is then applied to demodulate and filter out the carrier frequency of transmitted continuous wave. The baseband radar signal, *s*(*t*), can be written as [10]

(1) $$\begin{array}{c} s\left(t\right)=V_{0}+K\text{ cos}\left(\frac{4\pi }{\lambda }\left(d\left(t\right)+d_{\text{N}}\left(t\right)\right)\right)+w\left(t\right),\\ d\left(t\right)=d_{0}\text{ cos}\left(\theta_{\text{c}}\right)+d_{\text{C}}\left(t\right)+d_{0}\text{ cos}\left(\theta_{\text{a}}\right)+d_{\text{A}}\left(t\right)+d_{\text{H}}\left(t\right),\\ d_{\text{C}}\left(t\right)+d_{\text{A}}\left(t\right)=\left(r_{\text{c}}\text{ cos}\left(\theta_{\text{c}}\right)+r_{\text{a}}\text{ cos}\left(\theta_{\text{a}}\right)\right)\times \text{sin}\left(\omega_{\text{b}}t+\phi_{\text{0b}}\right),\\ d_{\text{H}}\left(t\right)=r_{\text{h}}\text{ cos}\left(\theta_{\text{c}}\right)\times \text{sin}\left(\omega_{\text{h}}t+\phi_{\text{0h}}\right), \end{array}$$

where *V*_0_ is the DC voltage, *K* is the gain of the radar, and *d*(*t*) is the distance of the subject from the radar at time *t*. Wavelength of the CW radar is *λ*=*C*/*f*_c_, where *f*_c_ is the frequency of transmitted signal and *C* is the speed of light. In (1), *d*_C_(*t*), *d*_A_(*t*), and *d*_H_(*t*) represent the periodic displacements of chest, abdomen, and heart, respectively. *d*_N_(*t*) denotes the random body movements that appear as phase noise in the received radar signal. *r*_c_, *r*_a_, and *r*_h_ are the amplitude of the displacement of chest, abdomen, and heart, *ω*_b_ and *ω*_h_ are the angular frequencies of breathing and heart beat, respectively. Also, *ϕ*_0b_ and *ϕ*_0h_ are the initial phase of periodic movements of breathing and heart at *t*=0. For the sake of simplicity, it is assumed that abdomen and chest are moving with the same rate and initial phase as mentioned in [26]. In addition, the white noise, *w*(*t*), is added to the received signal and (1) is written in terms of Bessel functions as described in the following equation:

(2) $$\begin{array}{c} s\left(t\right)=V_{0}+K\times \text{Re}\left[e^{\left(4\pi /\lambda \right)\left(d_{0}+d_{\text{N}}\left(t\right)\right)}\overset{\infty }{\underset{n=-\infty }{\sum }}J_{n}\left(\frac{4\pi }{\lambda }\left(r_{\text{c}}\text{ cos}\left(\theta_{\text{c}}\right)+r_{\text{a}}\text{ cos}\left(\theta_{\text{a}}\right)\right)\right)e^{in\left(\omega_{\text{b}}t+\phi_{\text{b}}\right)}\overset{\infty }{\underset{m=-\infty }{\sum }}J_{m}\left(\frac{4\pi }{\lambda }\left(r_{\text{h}}\text{ cos}\left(\theta_{\text{c}}\right)\right)\right)e^{in\left(\omega_{\text{h}}t+\phi_{\text{h}}\right)}\right]+w\left(t\right), \end{array}$$

where *J*_*n*_(*r*) is a Bessel function of the first kind and *e*^*ir*×sin(*ϕ*)^=∑_*n*=−*∞*_^*∞*^*J*_*n*_(*r*)*e*^*inϕ*^ with *J*_*n*_(*r*)=(−1)^*n*^*J*_−*n*_(*r*). From (2), it can be seen that the received radar signal is composed of multiple harmonics of breathing and heart rate as well as intermodulations of these harmonics with amplitude of *J*_*n*_(4*π*/*λ*(*r*_c_ cos(*θ*_c_)+*r*_a_ cos(*θ*_a_))) × *J*_*m*_(4*π*/*λr*_h_ cos(*θ*_c_)) and angular frequencies of (*nω*_b_+*mω*_h_). Depending on the sum of maximum displacements of chest and abdomen *r*_c_+*r*_a_, and the displacement of heart *r*_h_, after some *n* and *m*, the terms in (2) will become negligible.

In order to estimate the breathing rate from the received radar signal, the frequency where the magnitude of spectrum is maximum is found within the range of normal breathing. According to (2), the amplitude of this harmonic is *J*_1_(4*π*/*λ*(*r*_c_ cos(*θ*_c_)+*r*_a_ cos(*θ*_a_))) × *J*_0_(4*π*/*λr*_h_ cos(*θ*_c_)), when *n*=1 and *m*=0 for fundamental frequency. It is noted that the amount of displacement may change the amplitude of the Bessel coefficients and number of nonnegligible coefficients.

According to [27], movements of chest and abdomen (*r*_a_ and *r*_c_ in (1)) can change in the range of a few millimeters in quiet breathing to a few centimeters in deep breathing, depending on the age, sex, and posture of the subject under study.  Figure 2 shows how significant harmonics are affected by the amount of displacement of abdomen. The same effect can also be seen through different amount of movements of the chest. To depict Figure 2, (1) is used to simulate breathing movements, *d*_C_(*t*)+*d*_A_(*t*), and radar signal, *s*(*t*), where each row shows a different scenario. In all the cases, the operating frequency of the radar is *f*_C_=24 GHz, *r*_h_=0.1 mm, heart rate is 72 beats per minute and breathing rate is 18 bpm, the horizontal distance of the subject from the radar is *d*_0_=2.5 m, the distance between chest and abdomen is *d*_ca_=0.5 m, and the height of radar receiver (in Figure 1) is *H*=2 m. In addition, the maximum displacement of chest is *r*_c_=1 mm and maximum displacement of abdomen is 1 mm, 5 mm, 20 mm, and 50 mm from top to the bottom, respectively. White noise is added to the received radar signal with signal-to-noise ratio (SNR) of 20 dB. As observed from the right column of this figure, the strength of breathing harmonic at breathing rate is ((*ω*_b_ × 60)/2*π*) bpm and also the other significant harmonics are affected as the displacement of abdomen changes. Further investigation shows that the estimation (rate of the strongest peak at the range of breathing) can significantly be impacted by the noise.

Figure 3 shows the results of a simulation when Fourier transform is used for estimation, the breathing rate estimation is sensitive to the distance of the subject from radar *d*_0_ and the displacement of the chest. In this simulation, for two arbitrary distances, 100 noisy versions of the radar signal are generated using (1) and values given in Table 1. The frequency of strongest peak in the range of breathing (6 to 24 bpm) is taken as the estimate of breathing. For each distance (*d*_0_), the average of estimations *μ*_rate_est__ and 95% standard interval of these estimations [*μ*_rate_est__ − *Z*_*α*_*σ*_rate_est__, *μ*_rate_est__+*Z*_*α*_*σ*_rate_est__] are shown in Figure 3 for a range of displacements of abdomen, where *Z*_*α*_ is the *Z*-score of *α*=0.05. It can be seen from the figure that the width of standard interval of estimation highly depends on the displacement of body due to breathing and the distance of the subject from the radar. This shows that these two examples are selected to show that the estimation of breathing frequency using Fourier transform with a single-channel CW radar may be problematic. It is also noted that in Figure 3, only additive noise is considered, yet random movements of body may affect this estimation, even more dramatically.

The most common approach used in estimating breathing rate is the Fourier transform, which is mostly suitable to analyze stationary signals having the same frequency content over time. Most of the literature focuses only on choosing the peak of the spectrum within the breathing frequency range using the standard discrete Fourier transform. However, when random movements are present, peaks due to breathing frequency may not be prominent, and hence estimation may either be biased or totally wrong. In this work, modifications to the Fourier transform such as windowed Fourier transform, chirp Fourier transform, and micro-Doppler series acquired from the radar return are employed to estimate the changing frequency of signal over time.

## 3. Methods and Materials

### 3.1. Estimation of Breathing Rate Using Time-Frequency Analysis

The signal model described in (1) represents a nonstationary signal that can be analyzed in time-frequency domain by applying Fourier transform in sufficiently narrow time windows, where the signal may be assumed stationary [28]. For a given *s*(*t*), the windowed Fourier transform (WFT), *S*(*f*, *t*) is constructed as follows:

(3) $$\begin{array}{c} S\left(f,t\right)=\frac{1}{2\pi }\int_{0}^{\infty }\hat{s}\left(u\right)\hat{g}\left(f-u\right)e^{iut}du, \end{array}$$

where $\hat{s}\left(u\right)$ is Fourier transform of *s*(*t*) and $\hat{g}\left(u\right)$ is Fourier transform of the Gaussian window defined as

(4) $$\begin{array}{c} g\left(t\right)=\frac{1}{\sqrt{2\pi f_{0}}}\;e^{\left(-{\left(t/f_{0}\right)}^{2}\right)/2}, \end{array}$$

where *f*_0_ is a resolution parameter that identifies the trade-off between time and frequency resolutions. In order to estimate the changing frequency of signal over time, for each time sample *t*_*n*_, the frequency in which amplitude of *S*(*f*, *t*_*n*_) is maximum is found, i.e., dominant frequency at time *t*_*n*_. In this work, the sequence of these frequencies *ν*(*t*) is extracted from the radar signal over time. It is noted that when *ν*(*t*) is extracted from the range of normal breathing, it represents micro-Doppler frequency of the signal over time and is related to time-varying velocity of chest and abdomen.

At this stage, the phase of *s*(*t*) in the range of breathing frequency is calculated by setting *n*=1 and *m*=0 in (2) and is written as

(5) $$\begin{array}{c} \Phi_{\text{s},\text{Breathing}}\left(t\right)=\frac{4\pi }{\lambda }\left(d_{0}+d_{\text{N},\text{Breathing}}\left(t\right)\right)+\omega_{\text{b}}t+\phi_{\text{0b}}, \end{array}$$

where *d*_N,Breathing_ represents all random body movements having the same velocity unlike the breathing-related Doppler and thus is detected in the range of the breathing frequency. By definition, *ν*(*t*)=(Φ′(*t*))/2*π* [28], where Φ′(*t*) is the phase derivative of *s*(*t*) with respect to time *t*. The dominant frequency of *s*(*t*) in the range of breathing can then be written as

(6) $$\begin{array}{c} \nu_{\text{s,Breathing}}\left(t\right)=\frac{4\pi }{\lambda }\;d_{\text{N,Breathing}}^{\prime }\left(t\right)+f_{\text{b}}, \end{array}$$

where *d*_N,Breathing_′(*t*) denotes the speed at which the random body movements occur. Since 4*π*/*λ* is about 1000 for the radar in our experiments, very slow movements of body parts may give rise to high Doppler frequencies and thus may not be detected as a strong harmonic in the range of breathing. In view of this, *ν*(*t*) is assumed to be a linear combination of breathing rate and low-frequency harmonics of noise and random movements, and *f*_b_ can be estimated via calculating the mean of *ν*(*t*) over a specified time window of radar signal.

Figure 4 shows the micro-Doppler sequence extracted for the simulated radar signals shown in Figure 2. In simulations, *d*_N_ is not included assuming that random body movement is too slow to be detected at low frequencies of breathing range. Yet, additive noise *w*(*t*) is considered. From this figure, the average and standard deviation of the extracted sequences are found to be 17.15 ± 0.16 bpm, 17.60 ± 0.26 bpm, 17.23 ± 2.39 bpm, and 17.41 ± 0.7 bpm, from top to bottom, respectively. However, the dominant frequencies in the range of breathing in frequency domain (calculated from right column of Figure 2) are 17.81 bpm, 18.28 bpm, 6.56 bpm, and 17.81 bpm, respectively. The actual breathing rate for all these simulated signals is 18 bpm. These estimations indicate that the average of micro-Doppler sequence is a more accurate way of breathing rate estimation using a single-channel CW radar. In addition, it is observed from this figure that for the third simulated signal, where *r*_a_+*r*_C_=21 mm, the estimation in frequency domain is inaccurate since the harmonic of breathing is very weak. In this case, the standard deviation of the extracted micro-Doppler sequence is larger than the other cases. Thus, the standard deviation of the extracted micro-Doppler is used to calculate the confidence interval of estimation as a measure of confidence of the estimation in Section 3.3.

### 3.2. Constructing Bootstrap Resamples

It is noted that we are only interested in the dominant frequency at the range of breathing. However, estimation of this frequency is affected by random body movements and intermodulations amongst breathing frequency, heart rate and other frequencies related to body movements. The contributions due to body movements can be estimated via constructing the breathing signal based on the estimated breathing rate, subtracting it from the original radar signal and calculating the residual.

In order to examine how noise and intermodulations affect the estimation of micro-Doppler frequency, the bootstrap resampling method is employed. The bootstrap resampling was first introduced in [29] and has been modified and used in several applications since then. For instance, in [30], bootstrap has been used for confidence interval estimation using percentile-t method. It should be noted that the bootstrap method estimates the residuals and resamples it many times to build multiple noisy versions of the measured signal and calculates the confidence interval for each estimated parameter by assessing how noise distribution can affect the estimated parameter [31–33].

In our experiments, random body movements and intermodulations are hidden in the phase of the residuals. Thus, in order to make the bootstrap method resamples, the residuals are first calculated and the phase of the residuals is randomized to build multiple versions of possible random intermodulations and body movements. These noisy versions of residuals are referred as “surrogates” and have been introduced in order to build noisy versions of a signal with the same energy and frequency spectrum [34].

In order to calculate the residuals, for each time sample *t*, the frequency associated with maximum amplitude of *S*(*f*, *t*) is found, i.e., micro-Doppler frequency *ν*(*t*) at time *t*. The average of *ν*(*t*) is taken as the estimate of breathing as described in Section 3.1. In order to reconstruct the breathing component in the time domain, the phase and amplitude of *S*(*ν*(*t*), *t*) are obtained. The reconstructed signal is subtracted from the original one, where the remainder (residual) is related to radar reflections from other parts of body or signals related to intermodulations of breathing and heart harmonics. Accordingly, a bootstrap resample of the radar signal is built through reconstructing the residuals with randomized phase and adding them to the breathing component extracted from the signal.

In order to estimate the bootstrap statistics from the constructed bootstrap samples, micro-Doppler frequency of each bootstrap resample is estimated and Student's *t*_score_ is calculated (described in Section 3.3), with respect to the estimation calculated from the original signal [33]. In order to calculate micro-Doppler frequencies, WFT uses multiple windows of signal similar to the block bootstrap method [35–37]. WFT uses overlapping blocks of the signal with the same length and is desired for block bootstrap for time series as it results in lower variance in estimators [38]. In view of this, in this work, a double-loop bootstrap method is used in order to generate bootstrap resamples and provide bootstrap statistics with higher accuracies [39].

### 3.3. Estimation of Confidence Interval

In the following, different steps for estimating the confidence interval of breathing rate are presented.

1. A 15-second long radar signal *s*(*t*) is taken and preprocessed using a Butter-worth filter with cut-off frequencies of 0.05 Hz and 5 Hz.
2. Using the WFT method, time-frequency representation of *s*_F_(*t*) of the preprocessed *s*(*t*) is constructed. Micro-Doppler frequency over time *ν*(*t*) is extracted in the range of breathing [0.1 − 0.5] Hz. Breathing rate ${\hat{f}}_{\text{b}}$, i.e., the average of *ν*(*t*), is estimated and standard deviation of *ν*(*t*), $\hat{\sigma }$, is calculated.
3. Using phase and amplitude of *S*_F_(*ν*(*t*), *t*), the breathing model, $s_{\text{F}}\left(t,{\hat{f}}_{b}\right)$ in the time domain is constructed and sum of the components related to random movements and intermodulations, $\hat{\varepsilon }\left(t\right)$, is calculated.

(7) $$\begin{array}{c} s_{\text{F}}\left(t\right)=s_{\text{F}}\left(t,{\hat{f}}_{b}\right)+\hat{\varepsilon }\left(t\right). \end{array}$$

(4) A surrogate sample of ${\hat{\varepsilon }}^{*}\left(t\right)$ is obtained by randomizing the phase of $\hat{\varepsilon }\left(t\right)$ in the frequency domain and the residuals in time domain are reconstructed. A bootstrap sample of the radar signal is constructed as

(8) $$\begin{array}{c} s_{\text{F}}^{*}\left(t\right)=s_{\text{F}}\left(t,{\hat{f}}_{\text{b}}\right)+{\hat{\varepsilon }}^{*}\left(t\right). \end{array}$$

(5) The micro-Doppler frequency, *ν*^*∗*^(*t*) of *s*_F_^*∗*^(*t*) in the range of breathing is extracted. The bootstrap statistics for this particular bootstrap sample can then be calculated as

(9) $$\begin{array}{c} T^{*}=\frac{{\bar{f}}_{\text{b}}^{*}-{\hat{f}}_{\text{b}}}{\sigma^{*}}, \end{array}$$

  where ${\bar{f}}_{\text{b}}{}^{*}$ and *σ*^*∗*^ are the mean and standard deviation of *ν*^*∗*^(*t*).
(6) Steps 4 and 5 are repeated *B* times.
(7) The bootstrap estimates are sorted as *T*^*∗*1^ < *T*^*∗*2^ < ⋯<*T*^*∗B*^, and 100(1 − *α*)% confidence interval is computed as

(10) $$\begin{array}{c} \left(T^{*U}\hat{\sigma }+{\hat{f}}_{\text{b}},T^{*L}\hat{\sigma }+{\hat{f}}_{\text{b}}\right), \end{array}$$

  where *U*=*B* − [*Bα*/2]+1 and *L*=*Bα*/2.

## 4. Experiment Setup and Data Collection

The data in this experiment were collected in a simulated prison cell at Carleton University, Ottawa, Canada, after obtaining the appropriate ethics approval. The room measured 3.35 × 3.15 × 2.95 m, and radar was mounted 2.70 m above floor level in one corner, a tripod mounted camera was kept in an adjacent corner, a bed was present along one of the walls opposite to the radar, and a prison-type stainless steel toilet and sink (one joint structure) was kept close to the wall that was opposite to the radar (Figure 5). The radar used in this experiment was a 24.125 GHz CW single-channel Doppler radar prototype model built by K&G Spectrum in Gatineau, Canada, equipped with four adjacent transmit/receive antenna pairs each with 20 × 70 degree beamwidth. It should be noted that all four transmitter antennas simultaneously transmitted the signal and only one receiver antenna received it at any point in time. A Bosch NE1368 vandal-proof wide angle camera was also used in the experiments for recording baseline activity and posture information. The bed was constructed of concrete support blocks and oriented strand board, and a cotton filled mattress was placed on top of the board. The door of the room was closed, and only the test subject was present in the room. A Braebon model number 0528 piezoelectric respiratory effort sensor was fitted to the subject's chest at sternum level for monitoring breathing activity and three Ambu Blue-T ECG sensors were adhered to the subject's left and right wrists and left ankle for monitoring the ECG signal. All data were streamed to two computers situated outside of the room for recording. Radar data and ECG/breathing belt data were streamed via USB and Bluetooth, respectively, to Computer 1, and camera data were streamed via Ethernet to Computer 2. Three subjects, one male (22 years old, 164 cm height, 60 kg weight) and two females (24, 155 cm, 50 kg and 36, 160 cm, 70 kg), participated in data collection. The following test protocol was followed by all subjects with breaks in between each test:

1. Breathing normally and remaining still for 3 minutes:
  - Standing in front of bed and facing radar
  - Sitting on the edge of the bed and facing radar with hands resting on knees
  - Lying on bed in left lateral recumbent position and facing radar
2. Breathing normally and moving head shoulders and torso randomly for 3 minutes:
  - Standing in front of bed and facing radar
  - Sitting on the edge of the bed and facing radar with hands resting on knees
  - Lying on bed in left lateral recumbent position facing radar

A total 18 minutes recording for each subject was collected.

## 5. Results

As mentioned in [27], posture of the subject may have a substantial effect on the amount of movement of chest and abdomen. In this Section, three postures are investigated, namely, lying down, sitting, and standing, and the results are presented. In addition, the proposed method discussed in Section 3.3 is compared to the other breathing rate estimation methods using CW radar in the literature. In the ubiquitous method of estimating breathing rate, the frequency with the maximum energy (dominant frequency) in the frequency spectrum of the signal in the range of breathing is considered. In order to estimate breathing frequency, the signal is first preprocessed according to Step 1 of the proposed procedure described in Section 3.3. A Hamming window is then applied to the signal, and the chirp transform of the signal is obtained in the range of (0–4) Hz. It has been shown that the chirp transform results in more accurate estimations than regular DFT, since it benefits from improved frequency resolution in the range of frequency of interest [40, 41].

### 5.1. Lying Down

In the case of a lying down subject, it is observed for most cases that the breathing frequency estimated from the received radar signal is close to that obtained from the RIP signal and the number of significant harmonics related to random body movements or intermodulations is minimum.

Figure 6 shows 15 seconds of the recorded signal when Subject 1 is lying down on the bed, relaxing and breathing normally. It is observed from the RIP signal the subject's breathing pattern is regular and almost periodic. In this example, the radar signal is similar to RIP signal, similar to the simulated signal in the first row of Figure 2.

Figure 7 shows WFT as well as frequency spectrum of the radar signal. It can be seen from this figure that both Fourier transform and WFT exhibit a single significant harmonic at the rate of breathing. Micro-Doppler frequency of radar signal is the dominant frequency in the range of breathing, as shown in Figure 6. The average of micro-Doppler frequencies is calculated as 15.97 bpm and considered to be the estimation of breathing rate. It is noted that the breathing rate calculated from the frequency spectrum (Figure 7(b)) is 16.6 bpm. The micro-Doppler frequencies are extracted from the time-frequency domain using WFT, as shown in Figure 7(a), and then, the signal is converted back to the time domain in order to obtain the breathing model shown in Figure 6. Finally, the residual signal is calculated by subtracting the radar signal from its reconstructed version.

As discussed in Section 3, 200 bootstrap resamples of the signal are constructed. Micro-Doppler frequency of each bootstrap sample as well as the bootstrap statistic *T*^*∗*^ is calculated.  Figure 8 shows the density function of the bootstrap statistics obtained from 200 resamples. In this figure, *T*^est^=0 is the T-score related to the original signal, whereas *T*^*∗L*^=−0.44 and *T*^*∗U*^=0.27 specify the lower and upper limits of 95% confidence interval of this estimation, respectively. The confidence interval is estimated to be (15.5, 16.1) bpm. The reference breathing rate calculated from RIP signal is 15.6 bpm, and this, such a narrow confidence interval, confirms that the estimation is accurate.

### 5.2. Posture: Sitting

Similarly for the case of a subject sitting on a bed, breathing is regular, and the radar signal contains harmonics other than the breathing frequency. The time-frequency representation and frequency content of the radar signal are obtained. The dominant peak in the frequency domain is found to be 18.5 bpm. The sequence of micro-Doppler frequencies is then extracted from WFT, and their average is found to be 16.77 bpm. The residuals are then calculated, and its phase is randomized to generate a noise time series with the same energy. Finally, bootstrap resamples are constructed. The upper and lower bootstrap statistics are calculated as *T*^*∗L*^=−0.35 and *T*^*∗U*^=0.90, respectively, resulting in a 95% confidence interval of (16.3, 18.0) bpm, while the reference estimation calculated from RIP signal is 15.68 bpm.

### 5.3. Standing

When the subject is standing, the abdomen moves without any restriction which may have an influence on the magnitude of periodic breathing movement seen by the radar. In addition, while standing, the body slightly moves back and forth in order to keep the balance. In this case, the radar recording is very different from RIP signal. WFT and chirp transform of the radar signal are obtained, showing that the frequency content of the signal changes dramatically over time, and thus, a strong dominant peak may not be found in the range of breathing rate in the frequency domain. The breathing rate is estimated by extracting the micro-Doppler frequencies to be 14.73 bpm, while the estimation from frequency domain is 24 bpm. It is noted that the energy of residuals is much higher than that of the breathing signal, since it contains intermodulations of large movements of abdomen and the other body movements. The bootstrap statistics are calculated and the upper and lower limits of T-score are found to be *T*^*∗U*^=0.86 and *T*^*∗L*^=−0.18, respectively, resulting in a 95% confidence interval of (14.32, 18.63) bpm. The reference estimation calculated from RIP signal is 16.03 bpm.

### 5.4. Random Body Movements

Random body movements with linear velocity of *V* translate into Doppler frequency of 2*V*/*λ* in the received radar signal. For instance, if a part of body moves with the velocity of 0.1 m/s, it leads to a Doppler frequency of 16 Hz. In view of this, these movements may be ignored when looking at WFT of the radar signal in the range of breathing and may not affect the extracted micro-Doppler series.  Figure 9 shows the effect of random body movements in the radar signal. It is seen from this figure that the received radar signal is very different from the breathing signal, and random body movements are present as high frequency artifacts.  Figure 10 shows WFT and chirp transform of the radar signal. The peak of the signal in the frequency domain occurs at 21.8 bpm, while the average of micro-Doppler series extracted from WFT is 17.8 bpm. From these figures, it can be observed that random body movements give rise to very strong residuals. Phase of this residual signal is randomized to generate other possible random movements that could be added to the breathing signal. The bootstrap statistics are calculated and shown in Figure 11. The upper and lower T-score are calculated as *T*^*∗U*^=1.2 and *T*^*∗L*^=−1.3, respectively, resulting in 95% confidence interval of (14.40, 20.97) bpm. The reference breathing rate calculated from RIP is 16.03 bpm.

Breathing rate estimation results obtained using the proposed method as well as the reference value calculated from RIP and that obtained using the FFT-based method (estimated, actual, FFT) bpm, for three subject in three different postures, namely, lying down, sitting, and standing, are listed in Table 2.

It is known that breathing rate increases by age [42, 43]. From Table 2, the actual breathing rates for different postures show that the older subject have consistently higher breathing rate. It is also known that the breathing rate of overweight people is generally higher than the other people. Yet, the weight of all three subjects is considered normal and cannot be a discriminative feature in analyzing their breathing rate. In addition, women tend to breath faster than men [44, 45]. This is in accordance with the actual breathing rate of subjects. As seen from this table, the first two female subjects have higher breathing rates than the third (male) one. Height of the subjects has no considerable influence on their breathing rates.

### 5.5. Overall Results

Figure 12 shows the estimated breathing rate and confidence interval as well as the reference breathing rate calculated from RIP signal for a 6-minute experiment. In this experiment, the subject is lying down on a bed and stays stationary for the first 3 minutes. In the last 3 minutes, the subject moves her arms, head, and shoulders randomly. It is observed from this figure that estimated breathing rate matches the estimation obtained from breathing belt.  Table 3 summarizes all the estimation results. In this table, results are in the form of (mean ± standard deviation) of absolute errors between the estimated parameters and the reference estimation calculated from RIP signal. All the values are given in terms of breath per minute along with the number of outliers. It is noted that an element of a vector is called an outlier, if removing it decreases the mean of the vector by 5%.

In Table 3, breathing estimation obtained from chirp transform of the signal is compared with the average of micro-Doppler frequencies for different postures with or without random body movements. In all the cases, WFT is applied with *f*_0_=2. It is seen from this table that the accuracy of estimation is improved when using the proposed method instead of chirp transform of the signal. In other words, unwanted harmonics of the signal which are related to intermodulations between breathing and heart rate and also random body movements can affect estimation of breathing in frequency domain. However, when the signal is analyzed in time-frequency domain, harmonic of breathing can be separated from the other harmonics.

The most accurate estimation is obtained when the subject is stationary and lying down on a bed. In this case, even chirp transform results in an acceptable precision of measurement. Also, the estimated 95% confidence interval is very narrow (almost 1 bpm), indicating that we are quite confident about the estimated breathing rate and in 95% of cases, we would find the estimation in this range in presence of other sources of noise and body movements.

In the case of sitting, the estimation may be improved by using average of micro-Doppler frequencies instead of chirp transform. However, the 95% confidence interval is larger than that of the case, where the subject is lying down (3.05 bpm). In this case, slight movements of body due to balance may introduce uncertainty to the estimation. When the subject is standing, movements of body for balancing are larger and abdomen moves freely. In this case, chirp transform results in huge errors and, in some cases, the estimated breathing is twice that of the reference. Although the estimation improves to absolute error of 2.24 bpm using the proposed method, the width of confidence interval is 5.5 bpm, because of the significant energy of noise and unwanted harmonics with respect to the breathing harmonic.

When the subject starts moving head, shoulders, and torso, the accuracy of estimation using chirp transform drops severely. This estimation may be improved by using the proposed method. Yet, the confidence interval could be large indicating that these estimations are carried out in a noisy environment or in presence of random movements.

It is seen from the results that the proposed method is able to compensate for lack of quadrature channel and estimate breathing using single-channel CW radar with an average absolute error of estimation equal to 1.88 breaths per minute. Although this error seems high for monitoring patients, the error rate is satisfactory when the use of wearable devices or cameras is not allowed, such as continuous monitoring of breathing rate of inmates and elderly people, during sleep or rescue operations. It should be noted that breathing rate estimation is realized based on the detected motion, observed at a distance, and therefore is much more susceptible to noise, interference, and artifacts and is not expected to be as accurate at estimating breathing rate as the RIP band.

One of the limitations of the proposed method is that it is sensitive to the parameter *f*_0_ in (4), which controls the trade-off between time and frequency resolution of WFT. This parameter has been set to *f*_0_=2, which was found by trial and error and might need to be adjusted for other radar systems. In future works, ways of optimizing *f*_0_ needs to be investigated. The proposed method will also be examined in other environments where interference from other moving objects is present in the room.

It is noted that the system complexity, cost, and power consumption of a two-channel radar are well known to be higher than those of a single-channel radar, because a single-channel radar requires only one receiver branch [46, 47] and does not require balancing I/Q data [48].

## 6. Conclusion

In this work, a method for estimating breathing rate using a single-channel CW radar has been proposed. It has been shown through several simulations that Fourier transform-based estimation methods are not reliable to estimate breathing rate, when only one channel is used in the hardware of the radar. Quadrature receivers for vital sign monitoring have been well studied. However, single-channel receivers have not been well researched. Our study has demonstrated how single-channel radar can be used for monitoring in realistic situations and has provided estimates reasonably well. In case of a two-channel radar, the phase extracted from quadrature demodulation is a linear combination of breathing-related harmonic and those originated from noise and random body movements and can be processed by Fourier transform. However, in a single-channel CW radar, cosine of phase is received which is the output of a nonlinear system. In view of this, using time-frequency analysis has been proposed in order to extract the derivative of phase (or Doppler frequency) of the received signal over time. Using the proposed method, the received signal has been decomposed to the main harmonics originated from breathing and residuals, which are the sum of unwanted harmonics. Although the frequency of the main harmonic has been shown to be an estimate of breathing, our results have shown that this estimation can significantly be affected by unwanted harmonics. Therefore, bootstrap resampling has been used to support the estimations with a 95% confidence interval. Surrogates of unwanted harmonics have been generated by randomizing the phase of residuals, knowing that information of random body movements and unwanted intermodulations is hidden in the phase of the residuals. The results have also shown that the proposed method is able to compensate for lack of quadrature channel and can be used to estimate breathing using single-channel CW radar with an average absolute error of estimation equal to 1.88 breaths per minute.

## Figures and Tables

**Figure 1:** A subject is placed in front of the radar. Chest, abdomen, and heart move periodically.

**Figure 2:** Effect of displacement of abdomen on the strength of the breathing harmonic and the other nonnegligible harmonics in simulated radar signal. Values used for simulation are shown in Table 1, *r*_a_=1 mm, 5 mm, 20 mm, 50 mm from top to the bottom, respectively. (a) Breathing signal. (b) Radar signal. (c) Chirp transform of radar.

**Figure 3:** Estimated breathing rates vs displacement of the abdomen *r*_a_. Sensitivity of the estimated breathing rates to displacement of abdomen and distance of the subject from radar is shown, when Fourier transform of the signal is used to estimate breathing rate from noisy simulated signals (parameters are given in Table 1). (a) *d*_0_ = 2.5 (m). (b) *d*_0_ = 1 m.

**Figure 4:** Micro-Doppler sequence extracted for simulated radar signal shown in Figure 2.

**Figure 5:** Experiment setup.

**Figure 6:** From top to bottom: RIP signal, received radar signal, micro-Doppler frequencies extracted from WFT, breathing model, and residuals, when Subject 1 is lying down.

**Figure 7:** WFT and chirp transform of the radar signal, shown in Figure 6, when the subject is lying down on a bed.

**Figure 8:** Bootstrap statistics for 200 bootstrap resamples constructed from the radar signal shown in Figure 6.

**Figure 9:** From top to bottom: RIP signal, received radar signal, micro-Doppler frequencies extracted from WFT, breathing model, and residuals, when Subject 1 is sitting on the bed and moves head, torso, and arms randomly.

**Figure 10:** WFT and chirp transform of the radar signal, shown in Figure 9.

**Figure 11:** Bootstrap statistics corresponds to the radar signal in Figure 9.

**Figure 12:** Estimation of breathing within a 95% confidence interval for a 6-minute experiment, where the subject is lying down and stationary for the first 3 minutes and moves shoulders, arms, and head randomly in the last 3 minutes.

**Table 1:** Values used for simulation in Figures 2 and 3. It is noted that bpm stands for breath per minute.

Variable	*H* (m)	*d*_0_ (m)	Breathing rate (bpm)	Heart rate (beat/minute)	*r*_c_ (mm)	*r*_h_ (mm)	*r*_a_ (mm)	*d*_ac_ (m)	*λ* (mm)
Value in Figure 2	2	2.5	18	72	1	0.1	(1, 5, 20, 50)	0.5	12.5
Value in Figure 3	2	2.5	18	72	1	0.1	(1–50)	0.5	12.5

**Table 2:** Breathing rate estimation using the proposed method as well as the reference value and that of the FFT-based method (estimated, actual, and FFT) bpm, for three subjects in three different postures, namely, lying down, sitting, and standing.

	Lying down	Sitting	Standing
Subject 1 (36, 160 cm, 70 kg)	(15.85, 15.60, 16.68)	(16.77, 15.68, 18.52)	(14.73, 16.03, 23.78)
Subject 2 (24, 155 cm, 50 kg)	(13.88, 14.42, 13.78)	(14.63, 15.01, 15.19)	(15.10, 15.23, 19.14)
Subject 3 (22, 164 cm, 60 kg)	(14.67, 13.67, 14.36)	(13.94, 14.15, 14.38)	(15.20, 14.26, 18.38)

**Table 3:** Summary of results for different postures with or without random body movements.

State of the subject	Number of samples	Absolute error with respect to reference in bpm (number of outliers)				Width of CI in bpm (number of outliers)
		Chirp transform	Average of micro-Doppler	Lower limit of CI	Higher limit of CI	
Lying down and stationary	50	1.32 ± 0.79 (1)	0.82 ± 0.54 (0)	0.88 ± 0.61 (2)	1 ± 0.67 (1)	0.96 ± 0.67 (3)
Sitting and stationary	51	2.8 ± 2.55 (0)	1.25 ± 0.87 (0)	1.52 ± 1.37 (2)	1.76 ± 1.52 (0)	3.05 ± 2.81 (0)
Standing and stationary	51	4.36 ± 2.78 (0)	2.24 ± 1.39 (0)	2.90 ± 2.07 (0)	3.73 ± 3.28 (1)	5.50 ± 4.92 (1)
Lying down with movements	51	3.87 ± 2.07 (0)	2.05 ± 1.22 (0)	2.61 ± 1.96 (0)	2.65 ± 1.96 (0)	3.86 ± 3.03 (0)
Sitting with movements	51	4.57 ± 2.60 (0)	1.76 ± 1.30 (0)	4.23 ± 2.93 (1)	2.89 ± 2.65 (2)	6.35 ± 4.99 (2)
Standing with movements	51	3.99 ± 2.41 (0)	1.84 ± 1.32 (0)	3.29 ± 2.54 (1)	1.97 ± 1.60 (3)	5.26 ± 4.22 (0)

## Data Availability

The data used in the experiments will be made available online.
